The article "Effects of Coenzyme Q10 on the ratio of TH1/TH2 in Experimental Autoimmune Encephalomyelitis Model of Multiple Sclerosis in C57BL/6" was published in 2014. Journal: Iran Biomed J.

# Effects of Coenzyme Q10 on the ratio of TH1/TH2 in Experimental Autoimmune Encephalomyelitis Model of Multiple Sclerosis in C57BL/6

**DOI:** 10.6091/ibj.13362.2014

**Published:** 2014-10

**Authors:** Maryam Soleimani, Seyed Behnamedin Jameie, Mahmood Barati, Mehdi Mehdizadeh, Mahdieh Kerdari

**Affiliations:** 1 *Dept. of Anatomy, Faculty of Medicine, Iran University of Medical Sciences, Tehran, Iran;*; 2 *Dept. of Medical Basic Sciences, Faculty of Allied Medicine, Iran University of Medical Sciences, Tehran, Iran; *; 3 *Dept. of Pharmaceutical Biotechnology, Shahid Beheshti University of Medical Sciences, Tehran, Iran; *; 4 *Cellular and Molecular Research Center, *Iran University of Medical Sciences*, Iran*

**Keywords:** Experimental autoimmune encephalomyelitis (EAE), Multiple Sclerosis (MS), Coenzyme Q10 (CoQ10)

## Abstract

**Background:** Multiple sclerosis (MS) is known as a progressive central nervous system inflammatory disease. Certain factors, such as interleukins, inflammatory cells, and oxidative stress are supposed to involve in MS etiology. Because of the important role of oxidative stress, antioxidant therapy for MS has received more attention. Although coenzyme Q10 (CoQ10) acts as an antioxidant, there is a lack of enough research on its effects on MS. Therefore, the present research was designed. **Methods: **C57BL/6 female adult mice (n = 30) were used in this study. The animals were randomly divided into trial and control groups. To induce MS, routine procedure for experimental autoimmune encephalomyelitis (EAE) was used, and scoring was performed based on clinical signs. By detecting score one, CoQ10 administration was started (10 mg/kg/three weeks). By using ELISA and real-time PCR, the brain levels of TNF-, IL-10, IL-4, and IL-12 were studied. Statistical tests were used to analyze the data and the *P* value less than 0.05 was considered to be significant. **Results:** Clinical symptoms in EAE animals were significantly decreased (*P*<0.05) as compared to control ones. In addition, the level of the TNF- was significantly decreased following CoQ10 administration versus IL-10. The ratio of TH1/TH2 interleukins in treated animals was significantly less than that in non-treated animals (*P*<0.01). **Conclusion:** Our findings showed that CoQ10 is capable of suppressing the inflammatory pathway of MS.

## INTRODUCTION

Multiple sclerosis (MS) is the most important central nervous system (CNS) progressive immune-mediated disease. Epidemiological findings have shown that the incidence of MS dramatically has been increased; however, the reasons for such an increase are still unknown. It has been demonstrated that MS is mainly characterized by the infiltration of perivascular CD^4+^ T-cell and mononuclear cells that leads to demyelination of axonal tracks in the CNS [1]. The myelin proteins, including myelin basic protein, myelin proteolipid protein (PLP), and myelin-oligodendrocyte glycol-protein (MOG) are attacked and destroyed by T cells or other immune responses [2]. An immunohistochemical study has confirmed the presence of the pro-inflammatory cytokines (such as TNF-  and IL-12) in chronic MS plaques but not in the CNS of controls or in the peripheral blood mononuclear cells of MS patients [3]. The cytokines produced by activated CD^4+ ^T helper cells determine the onset or the progression of a disease. TH1 and TH2 cells as the main sources of cytokines are important regulators of immune response [4, 5]. TH1 cells secrete pro-inflammatory cytokines, such as IFN-γ, IL-12, and TNF-. However, TH2 cells release cytokines, such as IL-4, IL-5, and IL-13, which respectively activate macrophages to clear intracellular pathogens and aid in class switching of antibody and removal of extracellular infectious agents [6]. 

The article "Effects of Coenzyme Q10 on the ratio of TH1/TH2 in Experimental Autoimmune Encephalomyelitis Model of Multiple Sclerosis in C57BL/6" was published in 2014. Journal: Iran Biomed J.

Regarding the importance of the role of various types of IL in MS, the ratio or balance of TH1/TH2 has received more attention. Among the certain kinds of interleukins, IL-10, IL-4, IL-12, and TNF- are seemed to be more important in onset, severity, and progression of MS [6]. IL-10, which is produced by monocytes, macrophages, B cells, and TH2, not only inhibits the production of other cytokines such as IL-1 and TNF- but also ceases the proliferation of T cells [7]. It has been reported that IL-10 mRNA is continuously expressed throughout the course of experimental autoimmune encephalomyelitis (EAE) in *Swiss/Jackson Laboratory* mice immunized with PLP [8]. IL-4 also acts in the same way as IL-10 and inhibits the activation of TH1 cells. Some studies have shown that IL-4 is implicated as a suppressor cytokine in EAE. IL-12, which is critical for the differentiation of TH1 cells, has been found to be elevated immediately prior to the onset of disease in a monophasic EAE rat model as well as in a murine model [9, 10]. 

TNF- production is associated with TH1 response. It classically induces the activation of a variety of cell types and the expression of adhesion molecules, chemokines, and cytokines. The expression of TNF- was reported in EAE model of MS [11]. Kuroda and Shimamoto [12] showed that the injection of TNF- lead to the significant prolongation of clinical EAE and more severe cellular infiltration in the spinal cord. Regarding the importance of interleukins in the onset and the progression of disease, the inflammatory processes are characterized by leukocyte infiltrating play a crucial role in the pathology of the MS lesion mediated by the production of inflammatory mediators [13]. Excessive release of free radicals may also play an important role in MS pathogenesis and promote transendothelial leukocyte migration that leads to oligodendrocyte damage and axonal degeneration [14]. Free radicals, such as nitric oxide, reactive oxygen species, and/or reactive nitrogen species, which are produced by macrophages, microglia, and astrocytes, result in the damage of neurons, axons, myelin, and oligodendrocyte [15]. Based on these findings, it seems that other non-inflammatory mechanisms such as mitochondrial dysfunction may also contribute to MS neurodegeneration [16]. As the role of mitochondrial dysfunction and reactive oxygen species has been shown by a study [17], our recent therapeutic strategy has been focused on antioxidant. 

The article "Effects of Coenzyme Q10 on the ratio of TH1/TH2 in Experimental Autoimmune Encephalomyelitis Model of Multiple Sclerosis in C57BL/6" was published in 2014. Journal: Iran Biomed J.

Some kinds of antioxidants such as coenzyme Q10 (CoQ10) have been introduced during the last decades. CoQ10 is a vital mitochondrial electron transporter cofactor that acts as a potent antioxidant and, thus scavenging free radicals and inhibiting lipid peroxidation [18]. CoQ10 has also anti-inflammatory effects and protects neurons against apoptosis [19]. In 2010, Bessler *et al.* [20] reported that the CoQ10 could modulate cytokine production. To what extent the CoQ10 could influence the level of certain cytokines and the ratio of TH1/TH2 is the question of the present research. 

## MATERIALS AND METHODS

***Biological models.*** Adult female C57Bl/6 mice (n = 30, 10-12 weeks old, 18-20 g, Pasteur Institute of Iran) were used in this study. The animals were randomly divided into four groups of six mice, including EAE, EAE + CoQ10, EAE+ sesame oil, and control. All the procedures used in this study were approved by the Committee of Ethics in Animal Research of the Iran University of Medical Sciences (Tehran, Iran). 

***Induction of*** ***experimental autoimmune encephalo-myelitis*** ***. ***To induce EAE, the following routine procedures were used. Briefly, the animals were immunized by a solution containing 300 μg MOG (Alexis, Switzerland) in 100 μl PBS that emulsified by CFA (1:1 ratio) (Sigma-Aldrich, USA). On day 0, each animal received subcutaneously 200 μl (2 single shot) MOG-CFA emulsion into two sites of the upper flanks. Female mice were injected intraperitoneally with pertussis toxin (400 ng/mouse, Sigma-Aldrich, USA) 1 and 48 h after immunization. Mice were then weighted daily after immunization, and EAE symptoms were observed. 

***Clinical*** ***experimental autoimmune encephalo-myelitis*** ***score. ***To approve the onset and the stage of progression of the disease, the standard scoring system was used [21]. Based on this method of scaling, the clinical signs of no symptoms were assigned as 0, distal weak or spastic tail as 0.5, completely limp tail as 1, limp tail and hind-limb weakness as 1.5, unilateral partial hind-limb paralysis as 2.0, bilateral partial hind-limb paralysis as 2.5, complete bilateral hind-limb paralysis as 3.0, complete hind-limb as 3.5, unilateral partial forelimb paralysis as 4, and moribund and dead as 5 [22].

The article "Effects of Coenzyme Q10 on the ratio of TH1/TH2 in Experimental Autoimmune Encephalomyelitis Model of Multiple Sclerosis in C57BL/6" was published in 2014. Journal: Iran Biomed J.

***Coenzyme Q10 administration. ***The animals showed score 1 received i.p. injection of CoQ10 (Sigma- Aldrich, USA) at the dose of 10 mg/kg in 0.5 ml sesame oil for three weeks. The control animals, received only the sesame oil as a vehicle. 

***Tissue preparation and histological study. ***Perfusion and fixation by aldehyde solutions were performed transcardially via left ventricle. The animal brains were removed and post-fixed in the same fixative solution overnight and then exposed to tissue processing and finally paraffin embedding. By using a rotary microtome (Leica- rm2235, UK), coronal sections of 4 µ were prepared. To confirm the EAE model and also demyelination, myelin-specific staining (i.e. luxol fast blue) was used. The total surface of demyelinated regions was calculated by Infinity software (v. 4.6, Lumenera Corporation, Canada). Based on Allen Mouse Brain Atlas, 20 cross-sections of 4 µ thickness of corpus callosum per mouse were prepared and studied as above. 

**Table 1:** Mean ± SD of cytokines in trial and experimental groups

**TNF-**	**IL-12**	**IL-10**	**IL-4**	**Level of cytokines**
778.5333 ± 86.8344	786.3333 ± 137.07419	233.9400 ± 115.27928	146.8650 ± 9.95500	Control
948.8000 ± 30.0000	1003.6667 ± 245.02517	136.8367 ± 90.49804	147.5417 ± 28.52250	EAE
754.1300 ± 115.0362	1149.6667 ± 704.40424	319.8133 ± 100.04145	264.0000 ± 16.94000	EAE + sesame oil
731.4667 ± 51.3939	938.0000 ± 555.23328	642.5533 ± 153.26108	227.6433 ± 65.21032	EAE + CoQ10

EAE, experimental autoimmune encephalomyelitis

***Study of the level of cytokines.*** The animals were sacrificed by a lethal dose of ketamine (100 mg/kg) and xylazine (20 mg/kg). The brain tissue of animals was removed and rapidly transferred to liquid nitrogen. To homogenize the tissue, the solution containing 1× lysis buffer, 1 × Tris buffer saline 1% Nonidet P-40, 0.5% sodium deoxycholate, 0.1% SDS, and 0.004% sodium azide was combined with 10 μl phenylmethyl-sulfonyl fluoride solution, 10 μl sodium orthovanadate solution, and 10-20 μl protease inhibitor cocktail solution per ml of 1 × radioimmunoprecipitation assay (RIPA) lysis buffer mixed to prepare complete RIPA (Santa Cruze, USA). Three ml of complete RIPA/g of tissue brain homogenate were spun at 10,000× g at 4 °C for 10 min, and supernatants were collected and stored at -70°C. To determine the systemic concentration of cytokines, mononuclear cells from the spleens of immunized mice at a concentration of 2 × 10^6^ cells/well were incubated for 2 days in a total volume of 1.5 ml of RPMI-1640 supplemented with 10% FCS, 1% Lglutamine, 1% HEPES, 0.1% 2ME, and 0.1% penicillin/streptomycin. The cell super-natants were collected and assayed for the presence of cytokines. The concentration of IL-12, TNF-, IL-4, and IL-10 in the supernatants of brain extraction was assayed by using ELISA method. 

The article "Effects of Coenzyme Q10 on the ratio of TH1/TH2 in Experimental Autoimmune Encephalomyelitis Model of Multiple Sclerosis in C57BL/6" was published in 2014. Journal: Iran Biomed J.

***RNA extraction and real-time PCR. ***Animals were sacrificed by decapitation within a few seconds after being picked up from their home cage. The animal brains were removed and placed in sterile tubes, then freezed on dry ice. Total RNA extraction was performed using RNX-plus (CinnaGen, Iran). The RNA samples were re-suspended in 30 µl nuclease-free water. The concentration of total RNA was measured using a spectrophotometer (Pharmacia Biotech Ultrospec 3000, USA). The OD260/OD280 and OD260/OD230 ratios for RNA samples were 1.9-2.0 and up to 2, respectively. The first strand cDNA was synthesized with the First Strand cDNA Synthesis kit (Bioneer kit, K-2101, Korea). For each reaction, 1 µg RNA was used for reverse transcription in a mixture of 20 pmoles (1 µl) random primer and 18 µl DEPC-DW with a final volume of 20 µl. The mixture was incubated at 15°C for 1 minute, 50°C for 60 minutes, and heated at 95°C for 5 minutes to terminate the reaction. The cDNA was subsequently stored at -20°C. Real-time PCR was performed in a volume of 1 µl primer and 1 µl template plus 3 µl DEPC-DW with 5 µl Master mix (AccuPower® 2X GreenStarTM qPCR Master Mix, Bioneer kit, Korea). All PCR reactions were performed in the following conditions: started at 95°C for 15 minutes, followed by 40 cycles at 95°C for 15 s and 60°C for 30 s. The PCR primers for each gene are shown in Table 1. Each sample was tested in duplicate, and the values were normalized against the housekeeping gene, glyceraldehyde-3 phosphatede-hydrogenase (Table 2)*.*

***Statistical analysis.*** Data were analyzed and presented as mean ± SEM by using SPSS 21 and statistical exams. The result of the real-time PCR was analyzed by a two-sided student’s *t*-test. All mean differences were considered significant if *P*<0.05. Analyses were conducted using SPSS for Windows® v.21 (SPSS Inc., Chicago, USA).

**Table 2:** Nucleotide sequence of the forward and reverse primers for the real-time PCR

**Reverse primer-sequence (5´ to 3´)**	**Forward primer-sequence (5´ to 3´)**	**Target mRNA bases**
5’- GTCTTTGAGATCCATGCCGTTG -3’	5’- GCCCACGTCGTAGCAAACC -3’	TNF-
5’- TGGCCTTGTAGACACCTTGG -3’	5’- GCGCTGTCATCGATTTCTCC -3’	IL-10
5’- AAGCACCTTGGAAGCCCTAC -3’	5’- GTCACAGGAGAAGGGACGC -3’	IL-4
5’- CTGAGGACACATCCCACTCC -3’	5’- TGTCGCTAACTCCCTGCATC -3’	IL-12 subunit beta
CAACAATCTCCACTTTGCCACT -3’ 5’-	5’- TTGTGCAGTGCCAGCCTC -3’	GAPDH

GAPDH, glyceraldehyde-3 phosphatedehydrogenase

The article "Effects of Coenzyme Q10 on the ratio of TH1/TH2 in Experimental Autoimmune Encephalomyelitis Model of Multiple Sclerosis in C57BL/6" was published in 2014. Journal: Iran Biomed J.

**Fig. 1:** Luxol Fast Blue Staining. Significant differences are observed among different groups, including control **(A)**, EAE **(B)**, EAE + sesame oil **(C)**, and EAE + Q10 **(D)**. Demyelination area is shown by dots

## RESULTS

***Scoring.*** The scoring, which is considered as one of the important markers for the confirmation of EAE model significantly occurred in EAE-induced animals as compared to control and sham vehicle. The maximum mean score for the EAE + CQ10 animals (1.6 ± 0.54) was significantly (*P*<0.05) lower than that in EAE animals (2.5 ± 0.9).

***Histological study. ***EAE caused a significant demyelination in a certain area of the brain such as corpus callosum. The comparison of EAE group with EAE + CoQ10 group (42.56 ± 37.12% and 31.19 ± 39.14%, respectively) significantly showed less demyelination in the second group (*P*<0.05) (Fig. 1). The result from the animals that received only sesame oil (vehicle sham group) significantly demonstrated less demyelination compared and EAE and EAE + CoQ10 groups (*P*<0.05) (Fig. 2). 

***Cytokine analysis. ***The level of brain cytokines, including IL-12, TNF- (TH1), IL-10, and IL4 (TH2) was measured on day 21 post-immunization. The levels of TNF- and IL-12 were higher but not significant in untreated group compared to the control animals (Table 1). Our finding showed that CoQ10 administration in trial group significantly decreased the level of TNF- as compared to untreated animals (*P*<0.01) (Fig. 3). This finding is also the same for control animals (*P*<0.05) (Fig.4). In contrast, elevated level of IL-10 was found in treated animals compared to non-treated (*P*<0.001) and control ones (*P*<0.05) (Fig. 3). Regarding the level of IL-12 and IL-4, no significant difference was observed between untreated and control groups. The result showed that the ratio of TH1/TH2 in EAE animals was higher than that in sesame- and CoQ10-treated animals (Fig. 4).

**Fig. 2:** Histogram of demyelination in corpus callosum. A significant difference is observed among experimental autoimmune encephalomyelitis (EAE), EAE + sesame oil, and EAE + CoQ10. The difference between EAE + CoQ10 and EAE + sesame oil is not significant.

**Fig. 3:** Cytokine levels. IL-10 in experimental autoimmune encephalomyelitis (EAE) group was significantly decreased as compared to control; however, this level was increased in two other groups (EAE + sesame oil) and (EAE + CoQ10). The level of TNF-  was decreased after therapy by CoQ10. *P<0.0.5; **P<0.01

***Cytokine gene expression. ***Pro-inflammatory cytokine expression was analyzed using REST software (Qiagen, Germany) (Fig. 5). IL-12 mRNA and TNF- mRNA expression were increased remarkably in EAE model. There was no significant increase of IL-4 in anti-inflammatory cytokine mRNA expression in EAE as compared to control group. Although high increased expression of IL-10 mRNA did not occur in EAE animals, noticeable decline but not significant of IL-10 mRNA expression was seen in sesame and CoQ10 treatment groups. IL-4 mRNA expression in sesame oil group was obviously higher than control group, but IL-10 mRNA expression was obviously expressed lower in EAE mice. Also, a significant lower expression of TNF- mRNA was observed in animals treated with CoQ10 and sesame oils (Table 3).

The article "Effects of Coenzyme Q10 on the ratio of TH1/TH2 in Experimental Autoimmune Encephalomyelitis Model of Multiple Sclerosis in C57BL/6" was published in 2014. Journal: Iran Biomed J.

## DISCUSSION

In order to decrease or suppress the rate of MS progression, certain numbers of immunomodulatory and immunosuppressive agents have been used by various clinical disciplines. The role of interleukins in MS pathophysiology has been also reported by one study [13]. Clinical findings confirmed the serum alteration of IL-2, IFN-α (TH1), IL-10, and IL-4 (Th-2) in the patients with progressive MS and EAE model [7, 4]. IL-10 inhibits the production of several cytokines including IL-1 and TNF- and also decreases the proliferation of T cells [9]. Brosnan *et al.* [21] showed that the administration of anti-IL-10 monoclonal antibody in the murine EAE model worsen the rate of the disease. In 1998, Begolka *et al.* [22] demonstrated that IL-10 mRNA was continuously expressed throughout the course of EAE in *Swiss/Jackson Laboratory* mice immunized with PLP. It has been shown that IL-10-deficient C57BL/6 mice are more susceptible and develop a more severe form of EAE compared to IL-4-deficient mice [23]. Racke *et al.* [24] reported that i.p. administration of IL-4 reduced clinical severity of EAE. IL-4 mRNA was undetectable until the disease reduction in *Swiss/Jackson Laboratory* mice immunized with PLP [8]. However, little expression of IL-4 in the CNS has been found in other models of EAE [9]. Some studies have shown that IL-4 is implicated as a suppressor cytokine in EAE. Controversy about IL-4 still remains unsolved, and our data show unchanged level of IL-4 in EAE, although it was increased after treatment by CoQ10.

**Fig. 4:** Histogram of the TH1/TH2 ratio. Higher ratio is seen in experimental autoimmune encephalomyelitis (EAE( compared to other groups (*P<0.0.5).

The article "Effects of Coenzyme Q10 on the ratio of TH1/TH2 in Experimental Autoimmune Encephalomyelitis Model of Multiple Sclerosis in C57BL/6" was published in 2014. Journal: Iran Biomed J.

**Fig. 5:** The expression of mRNA. Using REST software, the fold changes were increased in inflammatory genes of EAE mice as compared to anti-inflammatory genes in this group (*P<0.0.5). BC, brain control

Regarding TNF-, it has been shown that mice transgenic for expression of TNF- lead to more oligodendrocyte apoptosis and demyelination [25]. This result approves the inflammatory role of TNF- and its expression that is parallel to the disease course [26]. Elevated serum of TNF- and peripheral mononuclear blood cells secreting TNF- have been reported in MS patients [27]. Kalman *et al. *[16] showed the functional involvement of mitochondrion in the development of MS. It has been demonstrated that any mitochondrial dysfunction results in a number of cellular consequences, including: decreased ATP production, increased reliance on alternative anaerobic energy sources, and increased production of reactive oxygen species [28]. Because most evidence has emphasized on inflammatory roles of cytokines in MS, using the anti-inflammatory drugs has received more application.

There are enough data suggesting that CoQ10 has beneficial effects on certain pathological conditions such as migraine, chronic tinnitus, hypertension, heart failure, atherosclerosis, age-dependent disorder, and cancer [29]. Regarding the effect of CoQ10 on IL-4, IL-10, IL-12, and TNF- in EAE, our finding is similar to different studies. For example, *Premkumar et al.* [30] reported that CoQ10 suppressed the production of inflammatory mediators such as IL-6 that is similar to what we found for TNF-. Following CoQ10 administration, IL-4 (TH2) remained unchanged but the expression of IL-10 (TH2) was increased significantly. Our result regarding IL-10 was similar to what reported by *Zhou et al*. [28] that confirmed the elevation of IL-10 in certain neurological disease. IL-10 (TH2) is able to inhibit synthesis of pro- inflammatory cytokines, such as IFN-γ, IL-2, IL-3, and TNF-, and thus promoting the survival of neurons and all glial cells [30]. IL-10 also limits inflammation in the brain via three major pathways, including reducing synthesis of pro-inflammatory cytokines, suppressing cytokine receptor expression, and inhibiting receptor activation [31]. Regarding the use of IFN-β, it has been approved that IFN-β helps to the balance or rebalance of the ratio of TNF- and IL-10 [27]. From this point of view, our findings clearly showed similarity therapeutic effects between using CoQ10 and IFN-β. How CoQ10 could act in the same way as INF-β is questionable and needs more future study. However, it has been shown that the beneficial clinical effects of CoQ10 could happen via different mechanisms. Among these mechanisms, immunomodulation properties of CoQ10 have received more attention. As mentioned previously, Fuller *et al.* [32] reported that CoQ10 could suppress the increased production of certain inflammatory mediators such as IL-6. In addition to the mentioned mechanism, it has been shown that CoQ10 inserts synergetic effects when combined with certain drugs in patients with cancer [30]. Administration of tamoxifen with CoQ10 in breast cancer reduces the time of treatment [33]. Restoration of a number of cultured damaged oligodendrocyte following the administration of CoQ10 has been reported by *Cammer *[34]. About the mechanisms, it has been generally accepted that CoQ10 not only produces sub-cellular energy but also acts as an antioxidant that prevents lipid peroxidation and scavenges superoxide anions [35]. CoQ10 can be diffused within biological membrane, and it can leak out the inner membrane of mitochondria [32]. N-acetyl cysteine, a known antioxidant, can block the effects of TNF- in HeLa cells. It acts via interaction with kinases involved in cellular signaling pathway [34]. Bessler *et al.* [19] reported similar result for inhibitory effects of CoQ10 on TNF-. It is possible that CoQ10 acts in the same way to block the effects of pro-inflammatory cytokines. Mao *et al. *[36] confirmed the effects of mitochondrial CoQ10, a derivative of coenzyme Q10, on EAE of C57BL/6 mice. They also explained that the mitochondrial CoQ10 inhibits neuronal loss via affecting the level of interleukins, such as IL-6, IL-10, TNF- etc. We believe that CoQ10 and mitochondrial CoQ10 may act in the same way [36]. Increasing the function of phagocytic cells, elevation of the level of the circulatory anti-inflammatory antibodies, preventing apoptosis are some postulated mechanisms for the role of CoQ10 [37]. Based on our findings, it is also possible that CoQ10 may act via involvement in regulating circulatory level of pro- or anti-inflammatory cytokines. 

The article "Effects of Coenzyme Q10 on the ratio of TH1/TH2 in Experimental Autoimmune Encephalomyelitis Model of Multiple Sclerosis in C57BL/6" was published in 2014. Journal: Iran Biomed J.

**Table 3:** Expression of mRNA analyzed by REST software

**TNF-**				**IL-12**				**IL-10**				**IL-4**			**Group**
**Result**	**P(H1)**	**Exp**		**Result**	**P(H1)**	**Exp**		**Result**	**P(H1)**	**Exp**		**Result**	**P(H1)**	**Exp**	
UP	0.004	6.052		UP	0.023	2.387		DOWN	0.045	0.589			0.682	0.831	Brain control- EAE
	0.317	1.31		UP	0	2.334		UP	0.01	1.803			0.056	2.136	Brain control-EAE + sesame oil
	0.056	1.561			0.862	1.037			0.121	2.014			0.566	0.831	Brain control-EAE + CoQ10
DOWN	0.018	0.258		UP	0.016	0.435		UP	0.034	3.416			0.976	1.000	Brain EAE- EAE + CoQ10
DOWN	0	0.217			0.914	0.978		UP	0.01	3.058		UP	0.041	2.571	Brain EAE- EAE + sesame oil
	0.189	1.556		UP	0.018	2.301			0.59	0.782			0.877	1.063	Brain oil-EAE + sesame oil
	0.091	1.583		UP	0.012	2.497			0.245	1.619			0.228	1.439	Brain Q10-EAE + CoQ10

Exp is related to mRNA expression, P(H1) shows P_v_, and Result is correlated with decrease or increase in gene expression. UP, up-regulation; DOWN, down-regulation

 With attention to immune-inflammatory basis of MS, the above mentioned mechanisms could explain the onset of MS. However, the continuation and progression of a disease is mainly neurodegenerative i.e. demyelination. The histological findings of our research confirm the findings reported by Kennedy *et al*. [38]. Altogether, it is logical that any therapeutic intervention could be able to cease or decrease the rate of first step of disease i.e. immunoinflammatory part, also might stop the later step or neurodegenerative part.
